The article "Serum Adiponectin Level in Different Stages of Type 2 Diabetic Kidney Disease: A Meta-Analysis" was retracted in 2023. Reasons: unreliable results or conclusions; concerns about the data; concerns about the results or conclusions; concerns about the peer review.

# Serum Adiponectin Level in Different Stages of Type 2 Diabetic Kidney Disease: A Meta-Analysis

**DOI:** 10.1155/2022/1863243

**Published:** 2022-07-15

**Authors:** Li Li, Jilai Shi, Guoliang Wu

**Affiliations:** ^1^Department of Endocrinology, The Affiliated Hospital of Shandong University of Traditional Chinese Medicine, Jinan, Shandong 250014, China; ^2^Department of Anorectal Surgery, The First Affiliated Hospital of Shandong First Medical University, Jinan, Shandong 250014, China

## Abstract

**Background:**

Biomarkers in predicting the stages of nephropathy associated with type 2 diabetes mellitus are urgent, and adiponectin may be a promising biomarker. This meta-analysis examined the association of serum adiponectin level with the stages of type 2 diabetic nephropathy.

**Methods:**

Databases including PubMed, Cochrane Library, EMBASE, China National Knowledge Infrastructure (CNKI), and Wan Fang were searched for published studies on adiponectin and type 2 diabetic kidney disease. The Newcastle-Ottawa scale was used to assess the quality of the literature. STATA 14.0 was used to conduct the statistical analysis.

**Results:**

Thirty-four studies with 5254 patients were included in this meta-analysis. The results of this study show that there was no significant difference in serum adiponectin level between normoalbuminuria and the control group (mean difference = −0.42, 95% CI [-1.23, 0.40]), while serum adiponectin level was positively correlated with the severity of type 2 diabetic kidney disease. The serum adiponectin level in type 2 diabetic kidney disease patients ranks as macroalbuminuria > microalbuminuria > normoalbuminuria.

**Conclusions:**

Serum adiponectin level might be an important marker to predict the progression of type 2 diabetic kidney disease.

## 1. Introduction

Hyperglycemia is the defining feature of diabetes mellitus (DM). Currently, DM is classified into two forms: type 1 (T1) and type 2 (T2) DM. T1DM is caused by the absolute lack of insulin which ensues consequent pancreatic beta cell destruction, while T2DM is mainly due to insulin resistance [1]. WHO reported that there were around 422 million people living with DM in 2018, and T2DM accounts for over 90% among these people [2]. Obesity is an important risk factor for T2DM [3]. The DM complications attack almost every body tissue, and DM is a leading cause of cardiovascular morbidity and mortality, blindness, renal failure, and amputations. Besides, the early diagnosis of T2DM in young people has been linked to a more aggressive form of the disease [4].

Long-term DM is closely related to microvascular complications, especially diabetic kidney disease (DKD). DKD is the most common complication of T2DM, which develops in around 40% of diagnosed patients [5, 6]. In addition, it is the leading cause of end-stage renal disease all over the world [7]. The definition DKD is based on current guidelines using four main criteria: a decline in renal function, proteinuria, and a reduction in glomerular filtration rate (GFR) [8]. DKD was divided into three stages according to albumin-to-creatinine ratio (ACR): normoalbuminuria (ACR < 30 mg/g), microalbuminuria (30 mg/g ≤ ACR < 300 mg/g), and macroalbuminuria (ACR ≥ 300 mg/g). It is crucial to diagnose patients who are more sensible to develop DKD for better control of the process of disease. Albuminuria has been one of the biomarkers to screen renal function; however, it has lots of limitations such as large variability and low sensitivity, and it may not be detectable in early stage [9, 10].

Biomarkers may allow earlier diagnosis and treatment for DKD, thereby slowing disease progression and raising life expectancy among patients [11]. Biomarkers are characteristic factors that can be measured and assessed as an indicator for normal physiologic or pathogenic processes. Examples of biomarkers are proteins, lipids, microRNAs, genomic, etc. Plenty of biomarkers associated with DKD were found in recent years, such as serum cystatin C, neutrophil gelatinase-associated lipocalin (NGAL), N-acetyl-*β*-D-glucosaminidase (NAG), and serum homocysteine (Hcy) [12].

Adiponectin (ADP) may play a role in DKD [13]. ADP is a small collagen-like protein expressed by adipocytes, which has been shown to have functions as anti-inflammation and insulin-sensitizing [14–17]. Reports of ADP effects on DKD have been variable; thus, a meta-analysis to obtain more precise evaluations is in need. This meta-analysis reveals the association between serum ADP levels and the severity of T2DKD. Results in this study may provide evidence to whether ADP can be a potential biomarker for DKD.

## 2. Methods

### 2.1. Data Source and Search Strategy

We identified studies published in PubMed, Cochrane Library, EMBASE, China National Knowledge Infrastructure (CNKI), and Wan Fang (last search date: April 24, 2022). The search terms included “adiponectin” and “diabetes mellitus” or “type 2 diabetes mellitus” or “type 2 diabetes” or “type 2 diabetics” or “ketosis-resistant diabetes mellitus” or “non-insulin-dependent diabetes mellitus” and “diabetic nephropathy” or “diabetic kidney disease” or “Kimmelstiel-Wilson disease”.

### 2.2. Data Extraction and Eligibility Criteria

Two investigators (Li Li and Guoliang Wu) independently extracted data and reached consensus, and the disagreement was determined by the third investigator (Jilai Shi). For each eligible literature, the following information was extracted: the first author's name, publication year, country, sample size, and data for ADP concentration.

Studies eligible for this meta-analysis should meet the following criteria: (a) the study included a control group (healthy people) and observation groups (DM patients with/without DKD); (b) observation groups including patients that were diagnosed as T2DM; (c) trials reported as RCTs (randomized controlled trials); (d) the literature reported the data for ADP concentration; (e) the literature was published in English or Chinese and the full text was available. Studies were excluded from our meta-analysis if they (a) did not report ADP concentrations in patients; (b) are animal or cell experiments, case report, review, letter, conference abstract, and those without full text; (c) are republished studies with similar data or patient; and (d) are irrelevant to the subject.

### 2.3. Quality Assessment

Quality of the studies included in this meta-analysis was evaluated by the Newcastle-Ottawa scale (NOS) assessment tool. These studies were judged based on three broad perspectives: selection, comparability, and exposure outcome. Studies with a score over 6 are considered of high quality.

### 2.4. Statistical Analysis

The relationship between adiponectin and diabetic kidney disease was reported as mean difference (MD) and 95% confidence intervals (CI) for continuous data using STATA 14.0 software (College Station, TX, USA). MD estimates were considered as significant if CI did not cross zero and *p* < 0.05. Pooled estimate was using a fixed-effect (absence of heterogeneity) or a random-effect (presence of heterogeneity) model. Heterogeneity between the studies was tested by *Q* test and *I*^2^ test. If *I*^2^ ≤ 50% or *p* (*Q* test) > 0.1, then no significant heterogeneity existed. Subgroup analyses were conducted to explore the potential sources of heterogeneity. Publication bias was assessed by Begg's test and funnel plot, and it was considered to be significant when *p* < 0.05. Pooled estimates were subjected to sensitivity analysis which involved excluding one study at a time and recalculating the summary effects to test the robustness of the results.

## 3. Results

### 3.1. Search Outcomes and Study Characteristics

Figure 1 outlines the study selection process in a flowchart following PRISMA guidelines. A total of 1638 literatures during the initial search were followed by omissions, and eventually, 34 studies were considered eligible and left for this meta-analysis.

The characteristics of the included studies are featured in Table 1. Overall, the total sample size included in this meta-analysis was 5254 with a wide range among patients across all studies (38 to 470). Of the included studies, 28 were conducted in China and published in Chinese, and the other 6 were conducted out of China and published in English. The mean NOS score was 7.15 ± 0.82, and all the included studies were of high quality with NOS scores above 6.

### 3.2. Meta-Analysis of the Relationship between Serum ADP and T2DKD

#### 3.2.1. Normoalbuminuria versus Control

In total, 31 studies were included in this meta-analysis, with 1354 healthy people and 1296 T2DM patients with normoalbuminuria. First, as depicted in Figure 2(a), there was a severe heterogeneity of these trials by comparing the MD of serum ADP (*I*^2^ = 98.5%, *p* = 0.001, random-effect model). The meta-analysis result indicates that there was no significant difference in serum ADP level between normoalbuminuria and the control group (MD = −0.42, 95% CI [-1.23, 0.40]). To explore the potential sources of the existed heterogeneity, subgroup analyses on sample size and nation (the study was performed in China or not) were performed. However, the heterogeneity still existed in either subgroup of sample size or nation (Figure 2(b)). Next, Begg's test was used to assess the potential publication bias. As shown in Figure 2(c), the funnel plot appeared symmetrical, and Begg's test result showed that no significant publication bias was in here (*p* = 0.959).

#### 3.2.2. Microalbuminuria versus Normoalbuminuria

In this meta-analysis, all the 34 trials were included, including 1337 patients with T2DM with microalbuminuria and 1438 with normoalbuminuria. As shown in Figure 3(a), a significant heterogeneity (random-effect model) existed with *I*^2^ = 97.8% and *p* = 0.001. Meta-analysis result shows that the level of serum ADP was higher in patients with microalbuminuria than those with normoalbuminuria (MD = 2.35, 95% CI [1.68, 3.02]). A subgroup analysis was also conducted here to find the potential sources of heterogeneity, and we found that the heterogeneity still existed in all the subgroups (Figure 3(b), sample size and nation). However, the combined effect changed in the large sample size subgroup (MD = 1.23, 95% CI [0.17, 2.64]) and the subgroup of trials that were not conducted in China (MD = 0.69, 95% CI [-3.07, 1.74]). As shown in Figure 3(c), the funnel plot appeared asymmetrical, and Begg's test result showed that there was a significant publication bias (*p* = 0.001).

#### 3.2.3. Macroalbuminuria versus Microalbuminuria

Similar results as *microalbuminuria* versus *normoalbuminuria* were found in this part. All the 34 trials were included in this meta-analysis, 1125 patients diagnosed as T2DM with macroalbuminuria and 1337 with microalbuminuria. As shown in Figure 4(a), a significant heterogeneity (random-effect model) existed here with *I*^2^ and *p* values of 98.0% and 0.001, respectively. In addition, the serum ADP level in patients with macroalbuminuria was higher than those with microalbuminuria (MD = 2.36, 95% CI [1.58, 3.14]). Subgroup analyses on sample size and nation did not eliminate the heterogeneity. However, the combined effect changed in the subgroup of trials that were conducted out of China (Figure 4(b), MD = 0.33, 95% CI [-0.80, 1.46]). Besides, the funnel plot of this meta-analysis appeared asymmetrical (Figure 4(c)), and Begg's test result showed that there was a significant publication bias (*p* = 0.001).

#### 3.2.4. Sensitivity Analysis

Since we found significant publication bias in the above studies (*microalbuminuria* versus *normoalbuminuria* and *macroalbuminuria* versus *microalbuminuria*), a sensitivity analysis was conducted by excluding one study at a time and recalculating the summary effects. As shown in Table 2, there is no obvious deviation or even reversal in the results obtained. The above data indicates that though significant heterogeneity existed in the study, the results are quite robust.

## 4. Discussion

T2DM accounts for more than 90% of all the DM patients worldwide. The complications of T2DM nearly affect all the body tissues, including kidney. It is worth noting that DKD is the most common complication of T2DM. Early diagnosis of DKD allows slow disease progression and relatively high life expectancy. Biomarkers provide the possibility for early diagnosis of DKD. ADP is a small collagen-like protein which has functions of anti-inflammation and insulin-sensitizing. Studies have shown that ADP may play a role in DKD; however, the relationship between them remains unclear and variable. Noel et al. [52] conducted a meta-analysis on this subject, and they had similar results as ours. They found that there is no significant difference in ADP levels between healthy people and DM patients with microalbuminuria. Besides, ADP levels were positively correlated with the severity of DKD. However, the amount of included studies was limited. Totally, 13 trials were included in their study, and only 6 of them were related to T2DM. In addition, Wang et al. [53] also performed a meta-analysis about this issue, and their findings were published in Chinese. In their study, 38 studies were included (both T1DM and T2DM) and all of them were conducted in China. Their results also reached a consensus that ADP levels were positively correlated with DKD severity. However, they pointed out the difference in ADP levels between healthy people and DM patients with normoalbuminuria which was not figured out in our study. Their results indicated that the concentration of serum ADP was higher in healthy people than normoalbuminuria DM patients (MD = −1.03, 95% CI [-1.76, -0.30]). The above reasons compelled us to conduct this meta-analysis.

In total, 34 trials with 5254 T2DM patients were included in this meta-analysis. The results of this study show that there was no significant difference in serum ADP level between normoalbuminuria and the control group (MD = −0.42, 95% CI [-1.23, 0.40]), while serum ADP level was positively correlated with the severity of T2DKD. The serum ADP level in T2DKD patients ranks as macroalbuminuria > microalbuminuria > normoalbuminuria.

The following are the limitations of this meta-analysis that should not be ignored. Most of the included studies were extracted from Chinese literature databases and were all published in Chinese. Though the other 6 literature were published in English, 5 of them were conducted in Japan, and thus, the quality of these trials remains doubtful. Besides, high heterogeneity and publication bias also brought limitation to the reliability of this meta-analysis. Fortunately, the sensitivity analysis indicated the robustness of our results. Based on the above reasons, more high-quality trials conducted and published in other countries are recommended in further evaluation.

## 5. Conclusions

In summary, our meta-analysis indicated that serum ADP levels were positively correlated with the severity of T2DKD. Therefore, serum ADP level might be an important marker to predict the progression of T2DKD. However, although quite a lot studies were included in this meta-analysis, heterogeneity and publication bias still existed, which affected the reliability of the results. Thus, more high-quality trials are recommended in further assessment.

## Figures and Tables

**Figure 1:** Flowchart of literature selection.

**Figure 2:** Meta-analysis of the relationship between serum adiponectin and type 2 diabetic kidney disease (normoalbuminuria *vs.* control): (a) mean difference of serum adiponectin level; (b) subgroup analysis; (c) publication bias.

**Figure 3:** Meta-analysis of the relationship between serum adiponectin and type 2 diabetic kidney disease (microalbuminuria *vs.* normoalbuminuria): (a) mean difference of serum adiponectin level; (b) subgroup analysis; (c) publication bias.

**Figure 4:** Meta-analysis of the relationship between serum adiponectin and type 2 diabetic kidney disease (macroalbuminuria *vs.* microalbuminuria): (a) mean difference of serum adiponectin level; (b) subgroup analysis; (c) publication bias.

**Table 1:** Characteristics of studies included.

Study	Year	Total sample size	Control			Normoalbuminuria			Microalbuminuria			Macroalbuminuria			NOS
			Sample size	Serum adiponectin		Sample size	Serum adiponectin		Sample size	Serum adiponectin		Sample size	Serum adiponectin		
				Mean	SD		Mean	SD		Mean	SD		Mean	SD	
Sun [18]	2021	226	60	15.10	1.20	74	12.90	1.40	66	8.70	1.70	26	4.50	1.90	7
Bai [19]	2019	190	50	3.19	1.26	61	4.25	1.33	44	6.34	1.27	35	13.41	2.62	8
Cheng [20]	2017	112	30	6.72	2.70	25	9.57	3.12	27	12.87	3.46	30	17.97	3.84	6
Xu [21]	2016	113	30	11.80	4.20	30	6.70	2.40	25	12.60	4.10	28	18.50	7.90	7
Tian [22]	2016	128	34	12.50	4.80	34	4.90	1.50	29	15.60	1.40	31	25.50	2.10	8
Bi [23]	2016	470	100	13.10	4.90	122	4.90	2.10	123	16.10	2.10	125	26.10	1.90	7
Zhou [24]	2015	172	85	73.40	9.90	37	39.40	13.50	30	54.40	10.20	20	67.80	11.30	6
Lu [25]	2013	258	62	10.22	2.13	62	8.55	1.86	70	5.93	1.64	64	3.58	1.37	7
Nie [26]	2012	140	35	9.72	4.30	35	3.27	0.68	35	10.88	2.85	35	12.75	2.46	8
Lin [27]	2011	200	50	9.58	1.33	50	16.88	1.77	50	22.54	1.86	50	28.12	2.11	6
Tang [28]	2011	132	35	12.70	5.00	35	5.10	1.70	30	15.80	1.60	32	25.70	2.30	8
Zhou [29]	2011	120	30	12.95	2.14	30	3.77	1.45	30	5.12	1.34	30	8.68	1.12	7
Hu [30]	2011	100	25	6.20	3.39	25	2.07	0.54	25	3.62	0.78	25	5.46	1.82	8
Wan [31]	2011	120	30	10.51	3.91	30	5.93	0.67	30	7.75	1.21	30	9.32	3.36	8
Xie [32]	2010	165	40	8.10	2.80	42	10.10	1.90	41	18.20	1.30	42	24.90	3.10	6
Li [33]	2010	220	51	9.69	1.26	67	16.92	1.36	57	21.34	1.67	45	26.21	1.95	8
Zhou [34]	2010	119	30	73.59	10.18	35	39.36	13.92	32	54.38	10.14	22	67.74	14.89	7
Zhong [35]	2010	130	45	5.63	1.16	25	6.28	1.87	31	9.28	2.59	29	11.15	3.18	7
Yang [36]	2010	150	40	5.15	1.99	40	10.12	1.70	40	16.58	2.68	30	7.40	1.28	6
Wan [37]	2010	130	30	11.20	3.50	36	3.40	0.80	34	9.60	2.20	30	14.30	5.60	8
Lin [38]	2010	120	30	6.44	3.11	30	2.21	0.55	30	3.62	0.80	30	5.31	1.86	6
Wu [39]	2009	151	47	10.10	1.82	32	16.41	1.94	40	18.32	1.30	32	25.52	3.19	7
Cheng [40]	2009	120	30	10.51	0.91	30	17.62	0.77	30	23.32	0.36	30	25.75	0.21	8
Yang [41]	2008	90	30	8.81	1.22	20	0.82	0.31	20	2.32	0.36	20	5.22	1.04	7
Liu [42]	2008	120	30	10.51	0.91	30	17.62	0.77	30	22.32	0.36	30	25.75	0.21	7
Yang [43]	2007	117	30	4.25	1.62	33	5.81	1.03	28	6.31	1.99	26	11.32	2.13	8
Zhu [44]	2007	213	50	14.69	7.12	52	7.78	3.55	57	10.15	5.83	54	153.98	6.33	8
Xiao [45]	2006	90	30	9.69	2.23	32	0.74	0.47	14	2.52	0.61	14	5.32	1.86	8
Kato [46]	2008	192	116	6.92	0.43	47	7.68	0.43	24	9.51	0.87	5	16.00	4.43	8
Yilmaz [47]	2008	123	N/A	N/A	N/A	38	24.10	6.10	40	16.80	2.70	45	13.30	3.10	7
Saito [48]	2007	259	49	8.99	1.12	76	6.38	0.56	106	7.67	1.25	28	5.75	0.97	6
Fujita [49]	2006	73	20	10.14	3.12	19	6.44	2.29	18	7.16	2.25	16	11.77	8.01	8
Komaba [50]	2006	153	N/A	N/A	N/A	86	7.08	5.47	44	10.65	6.07	23	14.14	8.71	6
Koshimura [51]	2004	38	N/A	N/A	N/A	18	6.50	2.10	7	7.90	3.80	13	11.00	5.50	6

Mean: *μ*g/ml; SD: standard deviation; N/A: not applicable.

**Table 2:** Sensitivity analysis.

Excluded study	Normoalbuminuria vs. control			Microalbuminuria vs. normoalbuminuria			Macroalbuminuria vs. microalbuminuria		
	*I* ^2^	*p*	Mean difference (95% CI)	*I* ^2^	*p*	Mean difference (95% CI)	*I* ^2^	*p*	Mean difference (95% CI)
Sun [18]	98.5%	0.001	-0.37 (-1.22, 0.47)	97.3%	0.001	2.50 (1.87, 3.12)	97.9%	0.001	2.50 (1.73, 3.27)
Bai [19]	98.5%	0.001	-0.46 (-1.30, 0.39)	97.9%	0.001	2.38 (1.68, 3.08)	98.0%	0.001	2.32 (1.54, 3.11)
Cheng [20]	98.5%	0.001	-0.46 (-1.30, 0.37)	97.9%	0.001	2.40 (1.71, 3.09)	98.1%	0.001	2.40 (1.60, 3.20)
Xu [21]	98.5%	0.001	-0.38 (-1.22, 0.46)	97.9%	0.001	2.37 (1.68, 3.06)	98.1%	0.001	2.41 (1.61, 3.22)
Tian [22]	98.5%	0.001	-0.36 (-1.19, 0.47)	97.8%	0.001	2.21 (1.55, 2.88)	98.0%	0.001	2.26 (1.48, 3.04)
Bi [23]	98.4%	0.001	-0.35 (-1.20, 0.49)	97.5%	0.001	2.25 (1.61, 2.89)	97.8%	0.001	2.26 (1.51, 3.01)
Zhou [24]	98.4%	0.001	-0.33 (-1.15, 0.50)	97.9%	0.001	2.39 (1.70, 3.09)	98.1%	0.001	2.40 (1.60, 3.21)
Lu [25]	98.5%	0.001	-0.40 (-1.26, 0.46)	97.5%	0.001	2.47 (1.81, 3.12)	97.8%	0.001	2.48 (1.70, 3.25)
Nie [26]	98.5%	0.001	-0.36 (-1.20, 0.47)	97.8%	0.001	2.31 (1.63, 2.99)	98.1%	0.001	2.42 (1.61, 3.23)
Lin [27]	98.3%	0.001	-0.59 (-1.38, 0.21)	97.8%	0.001	2.33 (1.65, 3.01)	98.0%	0.001	2.35 (1.55, 3.15)
Tang [28]	98.5%	0.001	-0.36 (-1.20, 0.47)	97.8%	0.001	2.23 (1.57, 2.90)	98.0%	0.001	2.28 (1.50, 3.06)
Zhou [29]	98.4%	0.001	-0.27 (-1.09, 0.55)	97.9%	0.001	2.40 (1.71, 3.09)	98.1%	0.001	2.35 (1.55, 3.14)
Hu [30]	98.5%	0.001	-0.37 (-1.21, 0.46)	97.9%	0.001	2.36 (1.67, 3.04)	98.1%	0.001	2.40 (1.60, 3.20)
Wan [31]	98.5%	0.001	-0.38 (-1.21, 0.46)	97.9%	0.001	2.37 (1.68, 3.06)	98.1%	0.001	2.43 (1.62, 3.23)
Xie [32]	98.5%	0.001	-0.46 (-1.30, 0.38)	97.8%	0.001	2.27 (1.60, 2.94)	98.1%	0.001	2.35 (1.56, 3.15)
Li [33]	98.3%	0.001	-0.62 (-1.40, 0.17)	97.8%	0.001	2.34 (1.65, 3.02)	98.0%	0.001	2.36 (1.56, 3.15)
Zhou [34]	98.5%	0.001	-0.34 (-1.17, 0.49)	97.9%	0.001	2.39 (1.70, 3.09)	98.1%	0.001	2.41 (1.60, 3.21)
Zhong [35]	98.5%	0.001	-0.45 (-1.29, 0.40)	97.9%	0.001	2.39 (1.70, 3.08)	98.1%	0.001	2.42 (1.62, 3.23)
Yang [36]	98.4%	0.001	-0.52 (-1.34, 0.29)	97.8%	0.001	2.34 (1.65, 3.02)	97.9%	0.001	2.55 (1.78, 3.31)
Wan [37]	98.5%	0.001	-0.32 (-1.15, 0.50)	97.8%	0.001	2.31 (1.63, 2.99)	98.1%	0.001	2.41 (1.60, 3.22)
Lin [38]	98.5%	0.001	-0.37 (-1.20, 0.47)	97.9%	0.001	2.36 (1.68, 3.05)	98.1%	0.001	2.41 (1.60, 3.21)
Wu [39]	98.4%	0.001	-0.55 (-1.35, 0.26)	97.9%	0.001	2.39 (1.70, 3.09)	98.1%	0.001	2.34 (1.55, 3.13)
Cheng [40]	98.4%	0.001	-0.69 (-1.49, 0.12)	97.8%	0.001	2.17 (1.50, 2.83)	98.0%	0.001	2.19 (1.42, 2.96)
Yang [41]	98.4%	0.001	-0.19 (-1.00, 0.62)	97.8%	0.001	2.29 (1.61, 2.97)	98.1%	0.001	2.32 (1.53, 3.11)
Liu [42]	98.4%	0.001	-0.69 (-1.49, 0.12)	97.8%	0.001	2.20 (1.54, 2.87)	98.0%	0.001	2.12 (1.35, 2.89)
Yang [43]	98.5%	0.001	-0.47 (-1.30, 0.36)	97.9%	0.001	2.42 (1.73, 3.11)	98.1%	0.001	2.36 (1.57, 3.16)
Zhu [44]	98.5%	0.001	-0.39 (-1.24, 0.46)	97.9%	0.001	2.42 (1.72, 3.12)	97.8%	0.001	1.91 (1.17, 2.65)
Xiao [45]	98.4%	0.001	-0.25 (-1.06, 0.56)	97.9%	0.001	2.32 (1.64, 3.00)	98.1%	0.001	2.37 (1.58, 3.17)
Kato [46]	98.4%	0.001	-0.49 (-1.32, 0.33)	97.9%	0.001	2.33 (1.65, 3.02)	98.1%	0.001	2.33 (1.54, 3.12)
Yilmaz [47]	N/A	N/A	N/A	97.9%	0.001	2.47 (1.81, 3.14)	98.0%	0.001	2.47 (1.68, 3.26)
Saito [48]	98.4%	0.001	-0.33 (-1.15, 0.50)	97.9%	0.001	2.40 (1.68, 3.11)	97.9%	0.001	2.48 (1.70, 3.26)
Fujita [49]	98.5%	0.001	-0.39 (-1.22, 0.45)	97.9%	0.001	2.42 (1.73, 3.11)	98.1%	0.001	2.42 (1.62, 3.22)
Komaba [50]	N/A	N/A	N/A	97.9%	0.001	2.41 (1.71, 3.12)	98.1%	0.001	2.43 (1.62, 3.24)
Koshimura [51]	N/A	N/A	N/A	97.9%	0.001	2.41 (1.72, 3.09)	98.1%	0.001	2.42 (1.62, 3.21)

Random-effect model used; N/A: not applicable.

## Data Availability

The labeled dataset used to support the findings of this study is available from the corresponding author upon request.
